# The Immediate Effect of Backward Walking on External Knee Adduction Moment in Healthy Individuals

**DOI:** 10.1155/2022/4232990

**Published:** 2022-11-11

**Authors:** Min Zhang, Jian Pang, Jiehang Lu, Meng Kang, Bo Chen, Richard K Jones, Hongsheng Zhan, Anmin Liu

**Affiliations:** ^1^Department of Orthopedics & Traumatology, Shuguang Hospital Affiliated to the Shanghai University of Traditional Chinese Medicine, No. 528 Zhangheng Road, Pudong New Area, Shanghai, China; ^2^University of Salford School of Health Sciences, Manchester, Salford M6 6PU, UK; ^3^Shanghai University of Traditional Chinese Medicine, Sports Department, No. 1200 Huatuo Road, Pudong New Area, Shanghai, China

## Abstract

Backward walking (BW) has been recommended as a rehabilitation intervention to prevent, manage, or improve diseases. However, previous studies showed that BW significantly increased the first vertical ground reaction force (GRF) during gait, which might lead to higher loading at the knee. Published reports have not examined the effects of BW on medial compartment knee loading. The objective of this study was to investigate the effects of BW on external knee adduction moment (EKAM). Twenty-seven healthy adults participated in the present study. A sixteen-camera three-dimensional VICON gait analysis system, with two force platforms, was used to collect the EKAM, KAAI, and other biomechanical data during BW and forward walking (FW). The first (*P* < 0.001) and second (*P* < 0.001) EKAM peaks and KAAI (*P*=0.02) were significantly decreased during BW when compared with FW. The BW significantly decreased the lever arm length at the first EKAM peak (*P*=0.02) when compared with FW. In conclusion, BW was found to be a useful strategy for reducing the medial compartment knee loading even though the first peak ground reaction force was significantly increased.

## 1. Introduction

The knee is one of the most important load-bearing joints during daily activities. During level walking, the forces across the knee are not distributed symmetrically between the medial and lateral compartments; rather, over 60% of the loading goes through the medial compartment of the knee. This asymmetry in the distribution of the force leads to a higher medial knee loading during gait [1]. Based on the finding previously reported, increased force is one of the potential contributing factors to the development and progression of some musculoskeletal diseases [2]. However, it is difficult to measure the loading at the knee during daily activities and it has been widely accepted that external knee adduction moment (EKAM) is a surrogate measure of the medial compartment load [3, 4].

A previous study indicated that every one unit (% Nm/Bw*∗*Ht) increase in EKAM would result in a reduction of 0.63 mm in the knee joint space width [5]. Moreover, a published report showed that every one-unit increase in EKAM is associated with a 6.46 times increase in the risk of progression of medial compartment knee osteoarthritis (OA) [6]. Therefore, reducing the EKAM has become the objective of gait modification in an attempt not only to reduce the medial knee loading but also to attempt in arresting disease progression [7]. In addition to EKAM, the knee adduction angular impulse (KAAI) has also been reported as a predictor of knee loading in the medial compartment [8, 9]. Moreover, some previous studies indicated that the KAAI is a more sensitive indicator than EKAM, as the first and second EKAM peaks during gait just represent the peak knee joint loading at the early and late stance phase, while the KAAI represents the entire loading in the medial compartment of the knee joint during gait [8, 9]. Therefore, it is important to include the KAAI in evaluating the loading of the knee during gait.

Backward walking (BW) has been reported as an effective rehabilitative exercise for improving the equilibrium of the human body, knee proprioception, and physical function [10–14]. It has been frequently recommended as a treatment for individuals who suffer from stroke, Parkinson's disease, and lower limb joint diseases [10, 12, 15]. Chen et al. [12] demonstrated that BW could significantly improve pain symptoms, physical function, and static stability in individuals with knee OA. Moreover, Gondhalekar and Deo [16] reported that BW could help to improve the clinical symptoms, knee joint range of motion (ROM), and hip abductor and extensor strength in individuals with knee OA.

Some previous studies indicated that the BW showed significantly higher first vertical ground reaction force (GRF) in the early stance phase, even though the walking speed in BW was statistically lower than that in FW [17–19]. The positive correlation between the first EKAM peak and first vertical GRF has been reported by some previous studies [20, 21]; therefore, the BW might lead to higher loading (EKAM) at the medial compartment of the knee during gait. However, no previous study reported the effects of BW on medial compartment knee loading during gait, and whether changes in walk direction could affect the EKAM and KAAI has not been studied. The aims of this study, therefore, were to investigate the effects of BW on EKAM in healthy adults. Since EKAM is the product of the GRF and the EKAM lever arm [22], this study also examined the changes in GRF and EKAM arms as secondary outcomes.

## 2. Methods

### 2.1. Participants

Twenty-seven healthy adults (15 men and 12 women) with a mean age of 25.04 ± 5.44 years, mean height of 1.69 ± 0.09 m, and mean body mass of 63.91 ± 12.81 kg participated in the present study (Table 1). Participants were recruited from the postgraduate students and staff of the Shanghai University of Traditional Chinese Medicine (SUTCM). Participants who met the following criteria were included in the study: (1) healthy; (2) 18 years and older; (3) no history of injuries to the lower limbs; (4) no disease or lower limb deformities that would affect gait patterns; (5) and able to walk without any assistive devices or aids. Participants who had any musculoskeletal or neurological disorders were excluded from the study.

Before formal data collection, the purpose of this study and the procedures involved were fully explained to each participant, and written informed consent was signed before their enrollment. Based on a statistical design, the sample size for this study was calculated using the software G*∗*Power (Version 3.1.9.6, University of Kiel, Germany), using an F-test statistical design (for EKAM) repeated measures with an effect size of 1.01 reported by a previous study, sample power of 95%, and an alpha value of 0.05. The analysis showed that a sample size of at least 9 participants would be suitable [3].

### 2.2. Ethics Statement

All experiments were approved by the China Ethics Committee of Registering Clinical Trials (ChiECRCT-20170066).

### 2.3. Instrumentation

The gait test was performed in the gait lab of Shuguang Hospital with a walkway of 8.6 meters long and 6.5 meters wide covered with a timber wooden floor. Retro-reflect marker's motion data were collected with the 16-camera VICON motion capture and analysis system (VICON, Oxford, UK) at a sampling rate of 100 Hz, The ground reaction forces were recorded with two 400 × 600 mm AMTI force plates (OR6-6, AMTI, USA) integrated and synchronized with VICON system at a sampling rate of 1000 Hz. To minimize the influence of footwear, all participants were asked to walk barefoot in BW and FW conditions.

Reflective markers (14 mm diameter) were attached to participants' specific bony landmarks (anatomical markers) according to a previously established model [23]. These were located at the anterior superior iliac spine (ASIS), posterior superior iliac spine (PSIS), iliac crest, greater trochanter, medial/lateral femur epicondyle condyles, lateral/medial malleolus, 1st, 2nd, and 5th metatarsal heads and calcaneus of both limbs. The markers placed on the anatomical landmarks were used to define the local coordinate system and joints center of each segment. Five rigid marker cluster plates with four noncollinear markers on each of them were used to track the movement of the pelvis, thigh, and shank segment and were fixed with an elastic bandage (Fabrifoam, USA) on the anterofrontal aspect of the bilateral shank, thigh and around the pelvis. The Calibrated Anatomical System Technique (CAST) was employed to determine the trajectory of these rigid segments and anatomical significance during the dynamic trials [24]. The test-retest reliability for measuring the variables of interest (i.e., 1stEKAM, 2ndEKAM, KAAI, and walking speed) in our lab was from good to excellent (intraclass correlation coefficient (ICC) of 0.83–0.95) in twelve healthy participants.

### 2.4. Data Collection

The VIOCN system was calibrated before the participants arrived. Upon the participants' arrival, the details of the experiment were explained, and consent forms were distributed and obtained after providing enough time for participants to think, ask questions, and decide. Before the formal gait test, participants' demographic characteristics (age, height, weight) were measured. Then, participants were asked to change into their shorts and a comfortable t-shirt. A static trial was performed for each condition before performing walking trials. Participants were instructed to walk backward with their head and upper body in a natural straight position. Both FW and BW trials were performed in one session. To reflect the natural stride length, the participants were asked to walk at their self-selected speed and comfortable pace. Moreover, the participants were asked to perform ten valid trials in each of the two conditions in a randomized order [17].

The sequence of FW and BW was randomly decided by asking participants to draw a card from a box; each card had a different sequence. Before formal data collection, each participant was given a few minutes for practice to get familiar with the way of walking and 20 minutes between conditions was given to allow participants to rest to minimize the fatigue effect. Considering the difficulties of BW and the possible fatigue effect on the biomechanical outcomes, participants were allowed to have a 20-second short break between trials. The kinematic and kinetic data were presented in a stance phase that was normalized to 100%. The data normalization has been added in the data results and analysis part. GRF was normalized to body weight and the EKAM was normalized to the participant's body mass.

### 2.5. Data Analysis

VISUAL 3D (Version 6.01.16, C-motion, USA) was used to calculate the kinematic and kinetic outcome measures. The kinematics data and analog data were filtered using a Butterworth 4^th^-order digital filter with a cut-off frequency of 6 Hz for the kinematics and 25 Hz for the analog data [24]. An inverse dynamics algorithm was used to calculate the primary biomechanical outcome, EKAM, and KAAI, in the stance phase for the trials at both BW and FW conditions. Based on a previous study [25], the quality checks were performed in Visual3D in order to avoid extreme kinetics and kinematics values. The EKAM and KAAI were normalized to the participant's body mass (Nm/kg and (Nm/kg)•s, respectively) and both the first and second peaks of EKAM were presented. The first EKAM peak was defined as the peak EKAM in the first half of the stance and the second EKAM peak was defined as the peak EKAM in the second half of the stance. The KAAI was defined as the positive area under the EKAM-time graph. The KAAI incorporates both the mean magnitude of the EKAM and the time for which it is imposed on the knee. The KAAI was calculated based on the EKAM and was presented with a unit of (Nm/kg) ·s, which was calculated by integrating the EKAM signal during a stance phase. The knee joint moment arms were defined as the perpendicular distance between GRF and the knee joint center in the laboratory frontal plane. Calculated at the time of the first and second EKAM peaks. Medial-lateral GRF was defined as a medial-lateral component of the GRF. The positive value is medial force. The early stance medial-lateral GRF was defined as the peak medial-lateral GRF in the first half of the stance and the second peak of medial-lateral GRF was defined as the peak medial-lateral GRF in the second half of the stance. Vertical GRF was defined as the vertical component of the GRF. The positive value is vertical force. The first peak of vertical GRF was defined as the peak vertical GRF in the first half of the stance and the second peak of vertical GRF was defined as the peak vertical GRF in the second half of the stance. The center of pressure (COP) was the distance of the center of pressure from the long axis of the foot (calcaneus to the 2nd metatarsal), where positive values indicate lateral. Calculated at the time of peak EKAM [26]. Based on a previous study, the quality checks were performed in Visual3D in order to avoid extreme data [25].

### 2.6. Statistical Analysis

The data from both legs were analyzed to satisfy the independence assumption of statistical analysis. Shapiro–Wilk tests were used to assess the normality of the selected parameters. The One-way repeated measure analysis of variance (ANOVA) was used to examine the difference in EKAM, EKAM arm, KAAI, GRF, and COP between FW and BW conditions. All statistical analyses were performed in SPSS (Version 16.0, IBM Corporation, USA) with a global alpha level of 0.05. For those variables that were significantly different between FW and BW, the relationships between their mean differences and mean difference in the first EKAM peak were evaluated using the Pearson *r* correlation coefficient [26]. Correlation coefficients were assumed very high when *R* > 0.8, high when *R* = 0.6–0.8, medium when *R* = 0.4–0.6, weak when *R* = 0.2–0.4, and very weak when *R* < 0.2 [19].

## 3. Results

The Shapiro–Wilk tests showed that both kinematic and kinetic parameters were normally distributed (*P* > 0.05). The biomechanical data in each condition are shown in Table 2.

A significant reduction in walking speed (1.30 ± 0.10 m/s, vs. 0.97 ± 0.13 m/s, *P* < 0.001) was observed in BW when compared with FW due to the invisibility of the direction of progress, however, the first peak vertical GRF in BW was significantly higher when compared with FW (*P* < 0.001) (Table 2, Figure 1). BW reduced the first EKAM peak, second EKAM peak, KAAI, first peak EKAM arm, and second peak vertical GRF significantly by 26.3% (*P* < 0.001), 16.0% (*P*=0.008), 16.7% (*P*=0.02), 40.0% (*P*=0.02), and 15.0% (*P* < 0.001), respectively (Table 2, Figures 1 and 2). Moreover, the medial-lateral GRF was found to act in the opposite direction in two conditions. For FW the medial-lateral GRF was positive, the GRF acted medially, while it acted laterally (negative) in BW (*P* < 0.001, Table 2, Figure 3). However, there was no significant difference in the second peak EKAM arm between FW and BW (*P*=0.25) (Table 2). When compared with FW, BW significantly shifted the COP medially at the time of the first EKAM peak (*P* < 0.001), and no significant difference in COP at the time of the second EKAM peak between FW and BW was found (*P* > 0.05) (Table 2). The relationships between mean change in variables that were significantly different between FW and BW in early stance and the first EKAM peak are reported in Table 3. Mean change in the first peak EKAM arm (*r* = 0.50), KAAI (*r* = 0.58), and COP at the time of the first EKAM peak (*r* = −0.43) was significantly covariate with the first EKAM peak (Tables 2 and 3). Thus, the first EKAM peak was strongly influenced by the first peak EKAM arm, KAAI, and COP at the time of the first EKAM peak. There was no statistically significant relationship between the mean change in walking speed (*r* = 0.04) and the mean change in the first EKAM peak (Tables 2 and 3). Thus, the first EKAM peak was poorly influenced by walking speed in this study.

## 4. Discussion

Some previous studies in BW focusing on lower limb joint diseases were performed on subjects with the specified problems [10–14]. However, the first vertical GRF in BW has been proven to be significantly higher in the early stance phase when compared with FW, even though the walking speed in BW was statistically lower than that in FW [17–19], which might lead to higher loading at the knee during gait. To date, no previous study reported the effects of BW on medial compartment knee loading during gait, and whether changes in the first peak GRF could affect the EKAM and KAAI has not been studied. Although there are indeed certain differences in biomechanical outcomes between patients and healthy individuals. This study was performed on healthy subjects because the outcomes would improve our understanding of the biomechanical impact of BW on knee loading, which has not been well-defined in previous studies. Therefore, no subjects with specified lower limb problems were employed for the study.

Our findings showed that BW significantly reduced the first and second EKAM peaks and KAAI. Such observations may be explained by the reduction of the EKAM arm caused by the opposite direction of medial-lateral GRF in early stance and the reduction of second peak vertical GRF during BW when compared with FW.

Compared with FW, the walking speed in BW was reduced by 25.3%. This finding was in accordance with a previous study that reported a 15.3% reduction in walking speed in BW [17]. This could be explained by a more cautious gait strategy due to the invisibility of the direction of the progress [27]. It was generally reported that decreased walking speed was associated with lower GRF during level-ground walking [28, 29]. However, the BW showed a larger first peak GRF during the early stance phase, which was similar to previous studies [17, 19]. The mean difference in walking speed and first peak vertical GRF were not significantly correlated with the mean difference in the first EKAM peak between FW and BW. This result indicated that the decrease in the first EKAM peak might not be dependent on the decreased first peak of vertical GRF caused by the reduction of walking speed. A similar finding has been reported by one previous study [19], which also demonstrated that the GRF peaks were poorly influenced by walking during BW. Moreover, we found the mean difference in the first peak EKAM lever arm was significantly correlated with the mean change in the first EKAM peak, which indicated that the reduction of EKAM was caused by the change in the EKAM lever arm. The second peak vertical GRF in BW was also significantly smaller than that of FW. These findings were similar to previous studies [17–19]. Since BW showed significantly higher first peak vertical GRF when compared with FW, the reduction of the first EKAM peak could be due to the shortening of the moment arm in BW, as the EKAM is mainly determined by the magnitude of GRF at the frontal plane (i.e., GF_frontal_) and the perpendicular distance (EKAM arm) between the knee center and the GRF vector [30].

Previous studies indicated that the EKAM arm reduction could be explained by the lateral shift of the COP due to the shortening of the perpendicular distance between the GRF vector and the knee joint center [31, 32]. However, BW showed a significantly smaller first EKAM peak even though the COP at the time of the first EKAM peak was shifted medially when compared with FW. The medial shift of COP at the first EKAM peak can be explained by the toe-contact to heel-contact during the early stance in BW [17], as a previous study indicated that the COP was shifted more medially during heel-off to toe-off in comparison with heel-strike to foot-flat in FW [13]. Since there was a significant medial shift of the COP in BW during the early stance, we suggested that other factors rather than the shift of the COP might have contributed to the decrease in the first peak EKAM arm in BW. We found that the magnitude of medial-lateral GRF in BW was quite different from that of FW. In FW, the magnitude of the early stance medial-lateral GRF was positive (medial direction) whereas BW showed negative early stance medial-lateral GRF (lateral direction) (Figure 3). This finding indicated that the direction of the medial-lateral GRF in BW was opposite to that of FW. The calculation of the frontal plane component of GF (i.e., GF_frontal_) was dependent on the GF_mediolateral_ and G⟶RF_vertical_ [30]. Due to the changes of GF_mediolateral_, the perpendicular distance between the knee joint center and the frontal plane component of GF_frontal_ was decreased (Figures 4 and 5), consequently, the EKAM arm was decreased so that the significantly smaller first EKAM peak was achieved in BW in comparison with that of FW, which was the real reason for EKAM reduction in BW. No significant difference in the second peak EKAM arm and the COP at the time of the second EKAM peak was found. However, the second EKAM peak was still significantly reduced by BW when compared with FW. This might be explained by BW significantly reduced vertical GRF by 15.0% in the second peak.

Additionally, the KAAI in BW condition was significantly reduced, which indicated that BW could not only reduce the EKAM peak, but also the whole loading of the knee during the stance phase. Previous researchers believed that the KAAI was more important than the peak value of EKAM, as it represents the resultant loading effect over the stance time in the medial compartment of the knee joint [8]. However, more studies concluded that the peak value of EKAM especially the first EKAM peak was strongly associated with the knee OA progression and was the main reason causing pain and damage to the knee joint [5, 33, 34]. Thus, the reduction in the EKAM peaks and KAAI in BW could be regarded as the positive outcome of the walking exercise for relieving the loading at the knee during gait.

EKAM peaks and KAAI were shown to be positively correlated with the development and progression of some musculoskeletal disorders such as knee OA [6]. The current study showed that BW could effectively reduce the EKAM peaks and KAAI. Therefore, we hypothesized that BW may be a useful strategy for individuals with medial compartment knee OA. With our preliminary findings among healthy young adults, such hypotheses should be tested in individuals with knee OA before conducting another randomized controlled trial.

There were several limitations in the current study. Firstly, only healthy young adults were recruited in the current study. Our findings should be further examined on the individual with medial compartment knee OA. Secondly, no surface electromyography (sEMG) data of the lower limb was included to identify the muscle activity in BW as previous studies have shown that muscle co-contraction influences knee joint compressive loading [35, 36]. However, healthy individuals are unlikely to have aberrant muscle co-contraction and thus this would be recommended in individuals with medial knee OA. Finally, lateral trunk lean was not measured and analyzed in the current study. Although in the protocol each participant was advised to keep their head and upper body in a natural straight position and both upper limbs waving in a natural way during the BW test. The effect of trunk posture on knee loading during gait in individuals with knee OA is critical [37]. Therefore, the outcome of lateral trunk leans during BW should be analyzed in the future.

## 5. Conclusion

The results of our study confirmed the significant biomechanical function of BW in reducing the knee joint loading, with the first and second EKAM peaks and KAAI decreasing significantly due to the change of the medial-lateral GRF and the reduction in the EKAM arm. We suggested that BW may potentially be a viable strategy in reducing medial knee loading for individuals with medial compartment knee OA.

## Figures and Tables

**Figure 1:** The vertical ground reaction force (GRF) during forward walking (FW) and backward walking (BW).

**Figure 2:** External knee adduction moment (EKAM) during forward walking (FW) and backward walking (BW).

**Figure 3:** The medial-lateral GRF during forward walking (FW) and backward walking (BW).

**Figure 4:** The illustration of the moment arm at the first peak of EKAM in forward walking (FW) and backward walking (BW), where *d* = EKAM arm.

**Figure 5:** Relationship between GRF_vertical_, GRF_frontal_, GRF_mediolateral_, and EKAM arm. The dashed arrow line represents the GF_vertical_, the dot arrow line represents the GF_frontal_, the solid arrow line represents the GF_mediolateral_, and the double solid line represents the EKAM arm.

**Table 1:** Characteristics of participants.

Sex	Male, 15/female, 12
Ages (years)	25.04 ± 5.44
Body height (m)	1.69 ± 0.09
Body mass (kg)	63.91 ± 12.81

**Table 2:** Comparison of biomechanical data between FW and BW (bold indicates significance).

Variables	FW	BW	Mean difference	*P* value
Walking speed (m/s)	1.30 ± 0.10	0.97 ± 0.13	−0.33 ± 0.11	**<0.001 ** ^*∗∗*^
The first EKAM peak (Nm/kg)	0.38 ± 0.13	0.28 ± 0.13	−0.09 ± 0.12	**<0.001 ** ^*∗∗*^
The second EKAM peak (Nm/kg)	0.25 ± 0.12	0.21 ± 0.08	−0.03 ± 0.09	**0.008 ** ^*∗*^
The first peak EKAM arm (m)	0.05 ± 0.04	0.03 ± 0.01	−0.01 ± 0.02	**0.02 ** ^*∗*^
The second peak EKAM arm (m)	0.03 ± 0.02	0.03 ± 0.01	−0.003 ± 0.02	0.25
KAAI (Nm/kg)•s	0.12 ± 0.06	0.10 ± 0.05	−0.01 ± 0.04	**0.02 ** ^*∗*^
Early stance medial-lateral GRF (body weight)	0.06 ± 0.01	-0.08 ± 0.02	−0.14 ± 0.03	**<0.001 ** ^*∗∗*^
Late stance medial-lateral GRF (body weight)	0.05 ± 0.02	-0.05 ± 0.01	−0.10 ± 0.03	**<0.001 ** ^*∗∗*^
The first peak of vertical GRF (body weight)	1.15 ± 0.09	1.32 ± 0.14	0.16 ± 0.13	**<0.001 ** ^*∗∗*^
The second peak of vertical GRF (body weight)	1.13 ± 0.08	0.96 ± 0.07	−0.19 ± 0.08	**<0.001 ** ^*∗∗*^
COP at the time of the first EKAM peak (mm)	7.73 ± 6.72	3.99 ± 5.72	−3.74 ± 9.00	**0.004 ** ^*∗*^
COP at the time of the second EKAM peak (mm)	7.66 ± 7.67	6.51 ± 6.19	−1.15 ± 9.47	0.37

^*∗*^ *P* < 0.05; ^*∗∗*^*P* < 0.001. Values were the mean ± SD. FW = forward walking, BW = backward walking, MD = mean difference, EKAM = external knee adduction moment, KAAI = knee adduction moment impulse, GRF = ground reaction force, and COP = center of pressure. A greater COP value refers to a more laterally located COP.

**Table 3:** Pearson's correlation coefficients (*r*) between the mean change in the first EKAM peak and mean change in other measured biomechanical variables.

Mean change in…	Mean change in the first EKAM peak (Nm/kg) Pearson *r*
Walking speed (m/s)	0.06
The first peak EKAM arm (m)^a^	0.50^*∗*^
KAAI (Nm/kg)•s	0.58^*∗*^
Early stance medial-lateral GRF (body weight)^a^	−0.001
The first peak of vertical GRF (body weight)^a^	0.18
COP at the time of the first EKAM peak (mm)^a^	−0.43^*∗*^

^*∗*^ *P* < 0.05. ^a^At time of first peak EKAM.

## Data Availability

The data to support the findings of this study are available from the corresponding author upon reasonable request.
